# Enriched Environment Regulates Dendritic Cells to Alleviate Inflammation in Cerebral Infarction Lesions

This article has been retracted.

**DOI:** 10.1155/2021/1574109

**Published:** 2021-12-24

**Authors:** Zhenzhen Zhong, Ping Xu, Jun Wen, Xiangdong Li, Xiaobo Zhang

**Affiliations:** Department of Neurology, The First People's Hospital of Changde City, Changde, Hunan, China 415000

## Abstract

**Objective:**

The aim was to investigate the role that enriched environment (EE) plays in the regulation of inflammation in cerebral infarction (CI) lesions and further explore the relationship between this regulation and dendritic cells (DCs).

**Methods:**

72 Sprague-Dawley rats were randomly divided into sham operation group (CON group, *n* = 24) and CI model group (*n* = 48). On completion of the establishment of CI rat models by Longa's method, rats in the models group were further assigned to standard environment group (NC group, *n* = 24) and EE group (*n* = 24). HE staining was utilized for evaluation of neuronal injury in the lesions. The number of CD74- and integrin *α*E-positive cells was detected by immunofluorescence. The expression of the IL-1*β*, IL-6, and TNF-*α* in the brain tissue and serum of rats was measured by immunohistochemistry and ELISA, respectively.

**Results:**

In comparison with the CON group, the NC and EE groups showed significant increases in neuronal injury, CD74- and Integrin *α*E-positive cells, DC content, as well as IL-1*β*, IL-6, and TNF-*α* expression in brain tissue and serum. According to the further comparison between the NC group and EE group, the latter showed decreases in each indicator, and these decreases were in a time-dependent manner.

**Conclusion:**

EE avoids the accumulation of DCs in the lesions and reduces the contents of IL-1*β*, IL-6, and TNF-*α*, consequently promoting the recovery of CI. And better recovery results can be obtained through increasing the time to stay in EE.

## 1. Introduction

An acute cerebrovascular disease known as cerebral infarction (CI) is associated with high incidence, disability rate, mortality, and recurrence rate [1]. Vessel occlusion is mentioned as the cause of CI, which results in decreased blood flow and, subsequently, ischemia and hypoxia in some brain tissues and, ultimately, necrosis of brain tissue [2]. CI is the second highest as shown in the published ranking of causes of death, and it is a major disabling disease worldwide [3]. Specifically, CI kills 2769 in 100,000 people per year, and three quarters of survivors have lost, in varying degrees, working capability, and becoming a burden to families and society [4]. Brain tissue injury after infraction is a complex process, which mainly includes direct injury of brain cells by ischemia and hypoxia, as well as indirect injury of brain tissue by inflammatory cells and a variety of inflammatory mediators [5]. Indirect injury, also known as secondary injury which is always induced by direct injury, is characterized by inflammatory cell infiltration (e.g., CD4 + T cells and NK cells) and cytokine (e.g., IL-6 and IL-1*β*) mediation [6]. Increased expression of cytokines such as IL-17, TNF-*α*, and IFN-*γ* in ischemic brain tissues has been mentioned by studies; elevated serum IL-6 and TNF-*α* levels mark cerebrovascular inflammatory damage and reflect proinflammation in CI patients [7]. Severe inflammation following cerebral ischemia in CI lesions is essential for CI, but its mechanism is yet to be elucidated in depth. We believe that studies on this mechanism can provide promising targets for the prevention and treatment of CI.

Dendritic cells (DCs) are the most potent antigen-presenting cells known to date, which enables the activation of immune response and the regulation of adaptive immunity [8]. The primary functions of DCs include antigen presentation, activating naive T cell, participating in the differentiation of T lymphocytes in the thymus, and inducing immune tolerance [9]. Particularly, DCs have a valuable function in neurological diseases, such as multiple sclerosis, Alzheimer's disease, CI, stroke, and epilepsy [10]. In patients with cerebrovascular stenosis, changes of the proportion of myeloid DCs (mDCs) in peripheral blood and mDCs decreased with the aggravation of cerebrovascular stenosis [11], suggesting that DCs are participants in the occurrence and progression of CI.

Enriched environment (EE) refers to a living environment of animals with advantages in terms of cage size and items placed in the cage, which is more conductive to increasing sensory stimulation, cognition, exercise, and social opportunities compared with the standard environment [12]. Numerous studies have confirmed that EE can cause morphological and structural changes in the nervous system and protect this system. And the promoting effect of EE on glial cell and oligodendrocyte regeneration in cortical areas, synaptogenesis, and angiogenesis and cortical thickness has been supported by the literature [13]. This indicates the importance and positive significance of EE intervention for ischemic CI. However, there is no literature confirming whether the regulation of DCs is involved in the mechanism by which EE attenuates inflammation of CI. Therefore, we carried out experiments for investigating how EE affected DCs in CI rats, thus clarifying that EE regulated DCs to reduce inflammation of CI and providing a new theoretical basis for treating CI.

## 2. Materials and Methods

### 2.1. Establishment and Grouping of CI Model

A total of 72 specific pathogen-free (SPF) Sprague-Dawley (SD) male rats weighing 180 ± 20 g were taken. Random grouping of the rats into 2 groups was conducted, namely, sham operation group (CON group, *n* = 24) and CI model group (*n* = 48). The CI rat model was established by common carotid artery (CCA) occlusion according to Longa's method [14]. Specifically, on completion of general anesthesia with 3% pentobarbital sodium (0.2 ml/100 g) under aseptic conditions, the right CCA, internal carotid artery (ICA), and external carotid artery (ECA) of rats were bluntly dissected. Then, the proximal ends of the ECA and CCA were ligated, the distal ends of the CCA were inserted a suture for further operation. Next, the ECA was cut to insert a suture, and the suture was inserted 10 to 11 mm into the ICA from the junction between ICA and ECA and subsequently fixed in the ICA. Finally, the wound was sutured, and the blood flow in the middle cerebral artery was successfully blocked. In contrast, rats in the CON group did not undergo ligation and insertion of the suture, while other procedures were the same as the model group.

The behavior of the rats was observed postoperatively. Successful modeling was indicated by the abduction and flexion of the left forelimb during lifting the tail, circling to the left and presence of Horner syndrome on the same side during crawling. Then, 24 h after modeling, based on evaluation of nerve injury by Zea-Longa score [15], rats with a score ≥ 2 was considered as successful CI models used for subsequent experiments.

After one day of CCA, CI rats were assigned to the standard environment group (NC group, *n* = 24) and the EE group (*n* = 24). Rats in NC group were housed in standard cages which were 25 cm × 20 cm × 20 cm with only food and water. EE housing includes a smaller cage (40 cm × 34 cm × 26 cm) and a larger cage (40 cm × 46 cm × 32 cm) connected by a circular tube (diameter: 7.5 cm, length: 20 cm). Inside the cage, there are swings, bowl-shaped running wheel, small houses, climbing ladders, colorful blocks, and so on [16]. In the EE group, toys with different shapes and colors in the cages padded with wood chips were replaced every 3 days, and the rats had free access to food and water. At 7 (*n* = 8), 14 (*n* = 8), and 21 (*n* = 8) days of feeding, serum was collected in each group by tail vein blood sampling, as well as brain tissue collection after euthanasia. This study was approved by the Medical Ethics Committee of The First People's Hospital of Changde City (2018-030-02).

### 2.2. HE Staining

The rats were anesthetized with 3% pentobarbital sodium (0.2 ml/100 g), and 4% polyformaldehyde was used and fixed in the rats. When the liver was fixed, the brain was taken and placed in 4% paraformaldehyde for 12 h. Subsequently, the embedded tissue samples were sectioned and rinsed three times with PBS. After 5 min staining with hematoxylin at room temperature, differentiation in hydrochloric acid alcohol and bluing in 1% (*v*/*v*) ammonia were followed. Then, after being washing with tap water, the sections were carried out eosin staining for 30 s, followed by dehydration with alcohol. The final step was to clear the sections with xylene and mount the sections. Observation of the pathological changes of brain tissues was completed under a microscope.

### 2.3. Immunofluorescence

After routine deparaffinization and rehydration, the sections were placed in 0.01 M citric acid buffer, followed by heat-induced antigen retrieval. Subsequently, they were soaked in a freshly prepared 3% H_2_O_2_-PBS solution for 30 min and then washed 3 times in ddH_2_O. On completion of the blocking step using 10% BSA dropped on the tissue, the sections were added with an appropriated amount of ddH_2_O and then were placed in an oven at a constant temperature of 37°C for 30 min. Subsequently, overnight incubation of the sections with primary antibodies CD74 and Integrin *α*E (1 : 100) was performed at 4°C, followed by rinsing step with PBS and another 30 min incubation with fluorescent secondary antibodies at 37°C.

After being rinsed with ddH_2_O for three times, 10 min incubation of the sections with ready-to-use DAPI at room temperature was carried out. The final step was to rinse the sections with ddH_2_O again and mount with antifade mounting medium. Photographs were taken using a microscope (CKX53, Olympus, Japan), and quantitative fluorescence analysis was performed utilizing Image J.

### 2.4. Immunohistochemistry

After deparaffinization and the rinsing step, the sections were placed in 10 mmol/l citrate buffer, boiled for 4 min, and then, removed. After washing with ddH_2_O and PBST, serum was utilized for blocking. Subsequently, primary antibodies diluted in 3% BSA-PBST were added for overnight incubation at 4°C. The sections rewarmed at room temperature for 60 min were carried out another 60 min incubation with enzyme-labeled secondary antibodies at room temperature. Finally, the sections were mounted, and a microscope was utilized for the observation of IL-1*β*, IL-6, and TNF-*α* expression in rat brain tissue.

### 2.5. Enzyme-Linked Immunosorbent Assay (ELISA)

Centrifugation of the rat serum collected from each group was carried out with the conditions of 200 g/min, 20 min, and 4°C, so as to remove cell debris. Then, the samples were placed into new EP tubes. Finally, measurement of IL-1*β*, IL-6, and TNF-*α* contents in rat serum was followed the instructions of the ELISA kits (Abcam, UK).

### 2.6. Statistical Analysis

SPSS 26.0 software was used for statistical analysis of the data. *T* test was used for comparison between the two groups, and one-way analysis of variance was used for comparison among multiple groups. Results were expressed as mean ± standard deviation (SD). A significant difference can be suggested if *P* < 0.05.

## 3. Results

### 3.1. Enriched Environment Reduces Cerebral Infarction-Caused Neuronal Injury

HE staining showed the normal neuronal structure and clear nucleoli in the CON group. In contrast, rats of the EE and NC groups had loose brain tissue on their infarcted side and decreased number of nerve cells. Disorganized cell structure, vacuolar degeneration of cells, nuclear lysis, and cell necrosis were the manifestations present in the latter two groups. Further, when compared with the NC group, the EE group had less neuronal injury and DCs, and degree of injury decreased along with the staying time in the EE (Figure 1). Collectively, EE contributed to the reductions in the CI-caused neuronal injury, and this reduction was time-dependent.

### 3.2. Enriched Environment Inhibits Cerebral Infarction-Caused Increases of Dendritic Cells

Subsequent immunofluorescence for determination of DC content in rat brain tissue showed that in marked contrast to the CON group, CD74- and Integrin ɑE-positive cells increased in the NC and EE groups, suggesting an increase in DC content. When compared with the NC group, significantly fewer CD74- and Integrin ɑE-positive cells, which indicated reduced DC content, presented in the EE group, and the cell number decreased along with staying time in the EE (Figures 2(a) and 2(b)). Collectively, EE could inhibit CI-caused increases of DCs, and this inhibitory effect was time-dependent.

### 3.3. Enriched Environment Reduces Cerebral Infarction-Caused Secretion of Inflammatory Factors

According to the immunohistochemical results, in comparison with the CON group, markedly increased IL-1*β*, IL-6, and TNF-*α* expression presented in the NC and EE groups. Further, when compared with NC group, the EE group had a reduction in the expression of these inflammatory factors, and this reduction was time-dependent (Figures 3(a)–3(c)).

According to the ELISA results, in comparison with the CON group, IL-1*β*, IL-6, and TNF-*α* levels in the serum significantly increased in the NC groups (*P* < 0.01). Furthermore, the concentrations of IL-1*β*, IL-6, and TNF-*α* were significantly lower in the EE group compared with the NC group, and the contents decreased with increasing time in the EE (*P* < 0.05; Figures 4(a)–4(c)).

Taken together, CI could promote the secretion of inflammatory factors in rat brain tissue and serum by CI, while EE could inhibit the CI-caused promotion, and this inhibitory effect was time-dependent.

## 4. Discussion

Normally, a few DCs exist in the meninges, choroid plexus, and cerebrospinal fluid, while after brain ischemia, DC markers (CD11c, MHC II) migrate into the ischemic lesion [17]. The involvement of DCs in acute CI and intracerebral hemorrhage has been supported by the literature. For example, infiltration of a large number of intracranial macrophages and DCs was found in the brain 12 hours after intracerebral hemorrhage [18]. And this infiltration of DCs has been confirmed to achieve through the peripheral circulatory system [19]. As proved by numerous studies, EE can cause morphological and structural changes in the nervous system and protect this system; regulation of damaged neurons by EE contributes to the promotion of postinfarction angiogenesis [20]. A consistent result was got by our research as by the report of Kostulas et al. [21] in determination of the accumulation of DCs in the ischemic CI lesions. We also found EE could slow this accumulation, and DCs in the lesions significantly reduced with increasing time in the EE.

CD74 can control myosin II to regulate actomyosin contractility and increase the ability of DCs to coordinate antigen processing and cell migration [22]; Integrin *α*E is a key protein for DC secretion and activation of inflammation in the body [23]. Through detecting the expression of CD74 and Integrin *α*E by immunofluorescence, we confirmed a significant reduction of CD74- and Integrin *α*E-positive cells in the EE group, and this reduction was time-dependent. Therefore, the conclusion that EE reduces the CI-caused accumulation of DCs can be obtained.

Some studies have confirmed that in cerebral ischemic tissues, cells in proinflammatory state produce a large number of inflammatory factors that cause a certain degree of damage to normal brain cells [24]. Moreover, these factors promote inflammatory cells to enter the immune response through the blood-brain barrier, thus directly or indirectly leading to brain tissue damage. Infiltration of large amounts of inflammatory cells and increased levels of inflammatory factors underlie the transition from cerebral ischemic damage to inflammatory damage, consequently contributing to the deterioration of the condition [25]. The involvement of DCs in brain tissue injury during CI has been reported to be achieved by releasing cytokines such as IL-6, TNF-*α*, and IFN-*γ* [26]. For reducing the inflammation in CI patients, an animal experiment has reported that EE, which provides tactile stimulation in many ways, can reduce TLR-2 content in brain tissue, thereby generally and continuously alleviating the inflammation in the brain of CI models and consequently improving the prognosis of the nervous system [27]. Another study also found that after being placed in EE for 14 days, CI rats showed the following changes: promotion of vascular endothelial cell proliferation, VEGF/Flk-1 expression, and cerebrovascular regeneration, while reduction of blood-brain barrier permeability and ischemia-reperfusion injury [28]. Collectively, EE can be predicted to slow CI-caused inflammation. For confirming this prediction, we herein measured the content of inflammatory factors in each group. The results revealed the ischemic CI-caused increases of IL-1*β*, IL-6, and TNF-*α* contents in the rat brain tissue and serum, while these inflammatory factors were appeared to decrease in the EE, and this decrease was in a time-dependent manner. In addition, studies have confirmed that EE plays a neuroprotective role by promoting neurotrophin expression and repairing astrocytes [29]. More specifically, EE can promote the enlargement of neuronal soma, reduce apoptosis, and cause morphological changes in dendrites, axons, and synapses. After the stimulation by EE, expression of nerve growth factor in animals marked increases, especially brain-derived nerve growth factor. Thus, it can be concluded that EE probably protects brain tissue by regulating DCs to inhibit the inflammation in the CI lesions.

## 5. Conclusion

In summary, EE avoids the accumulation of DCs in the lesions and reduces the contents of IL-1*β*, IL-6, and TNF-*α*, consequently promoting the recovery of CI. And better recovery results can be obtained through increasing the time to stay in EE. However, no studies have yet revealed the mechanism of EE regulating DCs. The confirmation of the relationship between the two can provide further understanding of the mechanism of EE protecting brain tissue, thus serving as a theoretical basis for the prevention and prognosis of CI.

## Figures and Tables

**Figure 1:** The enriched environment reduces neuronal cell damage caused by cerebral infarction (CI). HE staining was performed to observe the pathological changes in the brain tissue of each group of rats (scale bar = 50 *μ*M); per group *n* = 8. CON: sham operation group; NC: CI rats in the standard environment; EE: CI rats in the enriched environment.

**Figure 2:** Enriched environment inhibits cerebral infarction- (CI-) caused increases of dendritic cells. (a) Merge images of CD74 fluorescent antibody with DAPI staining; (b) merge images of Integrin *α*E fluorescent antibody with DAPI staining. Per group *n* = 8. Scale bar = 50 *μ*M. CON: sham operation group; NC: CI rats in the standard environment; EE: CI rats in the enriched environment.

**Figure 3:** Measurement of expression of IL-1*β* (a), IL-6 (b), and TNF-*α* (c) in rat brain tissue by immunohistochemistry (scale bar = 50 *μ*M); per group *n* = 8. CON: sham operation group; NC: CI rats in the standard environment; EE: CI rats in the enriched environment.

**Figure 4:** Measurement of the concentration of IL-1*β* (a), IL-6 (b), and TNF-*α* (c) in rat serum by ELISA. Per group *n* = 8; ^∗∗^*P* < 0.01 vs. CON group; ^#^*P* < 0.05 vs. NC group. CON: sham operation group; NC: CI rats in the standard environment; EE: CI rats in the enriched environment.

## Data Availability

The data used to support the findings of this study are available from the corresponding author upon request.
